# Research on Motion Behavior and Quality-of-Life Health Promotion Strategy Based on Bee Colony Optimization

**DOI:** 10.1155/2022/2222394

**Published:** 2022-03-04

**Authors:** Ruibi Chen

**Affiliations:** Wenzhou University of Technology, Wenzhou 325035, Zhejiang, China

## Abstract

Quality of life is a kind of sensory experience of people's physical health, social ability, and personal overall situation. Correct understanding and evaluation of the quality of life is conducive to human rational planning and control of life resources, promote physical and mental health, and improve the quality of life. In order to further explain the positive impact of physical exercise behavior on promoting physical and mental health, based on the bee colony optimization algorithm this paper analyzes the relationship between physical exercise behavior and quality of life and discusses the role of physical exercise behavior in promoting physical and mental health. The essential attributes and sociological significance of sports determine that sports play a unique role in providing people with social support. The quality of life score increases as the duration of the exercise increases. The theory and methods of defense and treatment advocated by sports thoughts will also have a positive effect on individuals avoiding and getting rid of mental illness. Teachers who have lower exercise time and frequency of exercise should also develop a step-by-step exercise program to strive to join them in the sports population.

## 1. Introduction

Quality of life is a kind of sensory experience of people's physical health, psychological function, social ability, and personal overall situation [1]. Sports can help the human body release excess energy, alleviate psychological pressure, reduce depression and anxiety, improve and regulate the psychological activities of modern people, enhance physical fitness and health, resist modern civilized diseases, alleviate subhealth status, and improve the quality of life of the sports population [2]. As an important index to evaluate the social development level of different countries, it is generally understood as the natural and social conditions of human existence. Quality of life is also a concept relative to the quantity of life. It is one of the comprehensive indicators for assessing the health level of individuals and groups and evaluating health promotion work [3]. Correctly understanding and evaluating the quality of life will help humans to rationally plan and control life resources, promote physical and mental health, and improve the quality of life. The bee colony optimization algorithm was chosen to analyze the correlation between health-related behavior and quality of life, allowing both independent and dependent variables to contain measurement errors [4]. Variables are not limited to a single indicator to measure and hence can be measured with multiple indicators. It is recognized that medicine should pay attention to the quantity and quality of life at the same time. The research work of quality of life is produced under this background and gradually developed and improved [5].

With the improvement of the level of science and technology and the development of modern civilization, the awareness of disease has also been improved by the extension of the average life expectancy of human beings. All of this has led to tremendous changes in human life and health views [6]. Quality of life is not only the goal of modern medicine but also an important step in health promotion and social diagnosis. Health-related behavior refers to behaviors related to health or disease in human individuals or groups [7]. People recognize that medicine should not only focus on the number of lives but also on the quality of life. The study of quality of life is produced in this context and gradually developed and improved [8]. Health-related behaviors can be divided into two categories according to the effects of behaviors on the health status of the actors themselves and others. They are promoting health behavior and endangering health behavior. Physical exercise is a physical activity in leisure time, which can help the human body release excess energy [9]. In order to make people aware of the promotion of sports on their quality of life, we conducted a questionnaire survey on sports and health knowledge, attitudes, beliefs, and behaviors of the people. The current situation and problems of quality of life and sports behavior were analyzed [10] to explore the methods and countermeasures of improving people's quality of life and physical exercise behavior.

The essence of sports is to promote people's physical and mental health development and improve people's quality of life by physical exercise as the basic means. Promoting health behavior refers to the behavior that is objectively beneficial to the health of individuals or groups. With the progress of human civilization, the improvement of living standards, the prolongation of life expectancy of the population, and the increase of the number of chronic patients, great changes have taken place in the outlook on life and health [11]. Sports are an important means to promote human health and enrich entertainment life. It is also an important symbol of humans' healthy and civilized life [12]. With the development of sports diversification and people's understanding of sports, physical exercise has become an indispensable part of our real life [13]. Through physical exercise, people can release stress and eliminate or alleviate negative emotions, thereby reducing the psychological burden of depression, autism, anxiety, etc., and thus playing a role in improving and regulating psychological activities [14]. The bee colony algorithm does not need to understand the special information of the problem. Through the local optimization behavior of each artificial bee individual, the global optimal value is emerged in the group, and the convergence speed is faster. Based on the bee colony optimization algorithm, this paper analyzes the relationship between physical exercise behavior and quality of life and discusses the effect of physical exercise behavior on promoting physical and mental health. It is expected to improve the people's sports cognition level and effectively guide them to develop healthy and reasonable physical exercise behaviors.

In this paper, we propose a research method based on bee colony optimization algorithm, which is a new algorithm for sports behavior and quality-of-life health promotion strategy research.

In summary, our contributions are as follow:

1. The bee colony algorithm makes the global optimal value emerge in the group through the local optimization behavior of each artificial bee individual
2. Based on the bee colony optimization algorithm, this paper proposes a new model for the relationship between physical exercise and quality of life
3. The technology has achieved better visualization effects in the research of health promotion strategies and effectively guides the people to develop healthy and reasonable physical exercise behaviors

## 2. Related Work

Physical exercise behavior is one of the main manifestations of human health-related behaviors. It is an objective and consciously controlled behavior of individuals or groups and an important means of promoting health [15]. Johannsen et al. believe that physical fitness behavior is a practical and conscious use of physical exercise means and methods and all practical activities carried out for the purpose of health [16]. Kretchmar believes that physical exercise is a kind of benign stimulation of various organs and systems in the body through scientific physical activity [17]. A series of adaptive reactions and changes occur in the body's morphological structure and physiological functions. Sports behavior is a kind of social behavior. It is an activity that human beings use various means and methods purposefully and consciously to meet certain sports needs. Dallat et al. combed articles published in the Journal of Psychological Research on the application of structural equation models and concluded that structural equation models have become an effective tool for psychological research [18]. Hawkes et al. made a comparative study on the health behavior disease cognition of different age groups. It was found that there were significant differences in health behavior among different age groups, and more health behaviors were taken with the increase of age [19].

## 3. Materials and Methods

Quality of life is a sensory experience that measures a person's physical health, mental health, social adaptability, and self-state. The evaluation of physical exercise behavior is a hot spot in international research. Studies have shown that physical exercise or physical activity includes factors such as work, life, and leisure. The relative contribution of physical exercise factors to the quality of life of people in different professional categories is clarified. The total quality of life is divided into dependent variables, and the scores of physical exercise are divided into independent variables [20]. Generally speaking, as the age of human beings grows, the functions of various organs in the body gradually decline, and chronic diseases increase. The adaptability to the environment, interpersonal, and other aspects has also begun to weaken, the physiological and psychological state has changed drastically, and the subjective life experience has begun to decline [21]. Quality of life is a multidimensional comprehensive measurement of the well-adapted state of the body, psychology, and society perceived by individuals or groups. Sports leisure consumption costs little or no consumption, most of the projects involved are simple, technical requirements are not high, the site requirements are not strict, and no capital investment is small. It means not only good health but also the value of life. The scores of emotional function and social function do not decrease with age, which indicates that the emotions of middle-aged college teachers are more colorful.

In order to improve the quality of life, we should not only strengthen our physique, improve our mental and physical health level, and prolong our life but also make our life fulfill its due responsibility and make its own contribution to the society and constantly improve its value. Colleges and universities should increase the propaganda of the benefits of physical exercise, while strengthening the teaching of physical exercise methods and means, and strive to popularize physical knowledge and exercise methods to every teacher. Both social environment and family environment provide adequate material and psychological support for their healthy growth. Once they leave the family and enter the university, the requirements for enjoying material life and improving learning conditions are relatively high. However, due to the existing conditions of the school, many of their psychological needs are difficult to meet. Teaching and educating people is a big systematic project. It is composed of subsystems such as party, government, industry, Youth League, teaching, scientific research, and logistics. Each subsystem is moving towards a common goal from different angles, cultivating socialist construction talents with ideals, morality, culture, and discipline. Therefore, we must coordinate and cooperate in many aspects in order to produce good effects. In the process of cooperation, teachers play a leading role, which is determined by the profession itself. Colleges and universities should not only create favorable conditions for teachers to learn sports knowledge but also regularly train college teachers in sports knowledge and sports skills and provide professional counselors at the same time.Physical activity and good living habits are the most active and economical means for us to maintain our own health and improve our quality of life. At any time, people must first meet the low-level physiological needs. Many manual workers often pursue high-level needs in their leisure time and pursue self-realization and self-worth and achievements.

Due to the limited training samples, appropriate compromises between generalization performance and recognition rate should be considered when determining nodes. The peak angles of the hips, knees, and ankles of the lower limbs of different sex subjects during jogging are shown in Table 1.

The establishment of the bee colony optimization algorithm model involves two problems, one is the parameter estimation of the model, and the other is the determination of the model order. Model parameter identification assumes that a data observation point is obtained. The model is

(1) $$\begin{array}{c} W=\gamma V\\ =\frac{\gamma IH}{\sin\;\alpha }. \end{array}$$

Then, complete the bee colony optimization operation as follows to take the criterion function:

(2) $$\begin{array}{c} \frac{{\text{d}}^{2}\omega }{\text{d}x^{2}}-\frac{h}{\alpha^{2}EI_{0}}\frac{\text{d}\tau }{\text{d}x}=-\frac{M}{EI_{\infty }}. \end{array}$$

Expand the above formula and apply the following vector differentiation formula:

(3) $$\begin{array}{c} B=\frac{Q}{\alpha Lh}\left[1-\frac{EI_{0}}{EI_{\infty }}\right]\tanh\frac{\alpha L}{2}. \end{array}$$

The estimated value of the parameter is obtained so that the output of the model best predicts the output of the system. Then, there are

(4) $$\begin{array}{c} \frac{{\text{d}}^{2}\tau }{\text{d}x^{2}}-\alpha^{2}\tau =-\frac{\alpha^{2}}{h}\left[1-\frac{EI_{0}}{EI_{\infty }}\right]V, \end{array}$$

(5) $$\begin{array}{c} C_{n}^{P}=\frac{\sum N_{S}^{P}n_{C}^{P}}{N_{S}^{P}}. \end{array}$$

The changes in the three-dimensional motion angle and muscle force of the knee joint in each analysis step were applied as a boundary condition to the finite element model. The motion angle parameters applied to the finite element model are shown in Table 2 and Figure 1. The relationship between the parameters of the lower rotation angle and the time in the case of the healthy side and the affected side is shown in Table 3 and Figure 2.

Physical education, with its special form of activities, rich activities, and the characteristics of different activities combining physical strength and intelligence, determines the interrelationship between physical exercise and health promotion. The commonality of physical labor and physical exercise is the energy expenditure of muscle activity, biochemistry, and substance catabolism. The school's public gymnasium is fully equipped, has a large space, and has many optional exercise programs and a comfortable environment. Many college teachers live near the school, so the school public fitness venue is the first choice for college teachers to participate in exercise [22]. If the amount of physical activity is too large, energy and material consumption, physical reserves are reduced, and the rest time is long, the body must need energy supplement and necessary anabolism, so rest and rest are understandable. With the rise of the sports industry, many exercise items and equipment are suitable for families, and exercise methods can also be learned from television and the Internet. At the cultural level, people are relatively closed and conservative, dependent and conformist, utilitarian pursuit, and experiential thinking. It all determines their behavioral patterns.

Most physical exercises require participants' physical and psychological activities to be in a certain state of excitement and activation. This is conducive to the improvement of health quality, emotional communication, and the elimination of self-claustrophobia. The indexes in the excessive recovery period were all restored to above the conventional level. The comparison of anaerobic power data before and after excess recovery is shown in Figure 3.

## 4. Result Analysis and Discussion

The human body is a very complex multi-degree-of-freedom motion system. It is very difficult to simulate the actual situation of the human body during exercise. The use of biomechanical knowledge in the daily physical training process is equally important. A competent sports instructor must be proficient in sports physiology and biomechanics. The lag of the development of social sports, the lack of investment in sports, the lack of interest in sports, and the lack of venue equipment and social guidance personnel are all important factors that restrict the participation of college teachers in physical exercise. For people, the greater impact on quality of life is behavioral cognition, behavioral habits, emotional experience, and behavioral control [23]. The effect of physical exercise is a gradual accumulation process, not once and for all. The health effect and physique enhancement of people's physical exercise are influenced by exercise prescription. The effects of physical exercise with different intensity on people's health physiology, psychology, and social health and physique enhancement are significantly different.

In the process of practical reform and practice, we must always take physical fitness as the main line of development and actively carry out sports training suitable for social needs. Blood ALP data before and after recovery are shown in Figure 4.

If it is recognized that the behavior of the monitoring object triggers the preset rule, the system automatically alarms. The subject's myocardial function has been enhanced, the heart's pumping function has been improved, and it is able to quickly adapt to the immediate heart rate after exercise and reduce the time required for recovery after exercise. The time is shown in Figure 5 when the subject's heart rate returns to a quiet heart rate immediately before and after the experiment.

Sports biomechanics will enable sports coaches to have a better understanding of the rules of biological movement, the interactions that affect biological movements, and the state of stress on joints during human movement. Randomly select input and output data and submit it to the network. Calculate the output of each neuron in the hidden layer:

(6) $$\begin{array}{c} W=\chi \frac{QL^{3}}{EI_{\infty }}+\Delta \kappa \frac{Q}{EI_{\infty }}. \end{array}$$

Calculate the response of the output layer neurons:

(7) $$\begin{array}{c} \underset{x}{\min}\sum_{\left(i,j\right)\in Lreal}\int_{0}^{x_{ij}}t_{ij}\left(\omega \right)\text{d}\omega . \end{array}$$

Calculate the error of the output layer neurons using the given output data:

(8) $$\begin{array}{c} CP\;D=\sum \frac{\left|\Delta \varepsilon_{pi}\right|}{\varepsilon_{y}}. \end{array}$$

Calculate the generalization error of each neuron in the hidden layer:

(9) $$\begin{array}{c} P_{s}=\exp\left[-{\left(\frac{\sigma }{\sigma_{0}}\right)}^{m}\right]. \end{array}$$

The pseudo-color editing of the moving image sequence is superimposed on the image monitor. Time-varying parametric curves and statistical results are obtained as output.  Figure 6 is the data of maximum motor ability before and after experiment restoration.

The essential attributes and sociological significance of sports determine that sports play a unique role in providing people with social support. Educational exercise is carried out through the interaction of people in the stadium, and this kind of interaction often appears in the form of groups. Health promotion refers to the process of improving people's physical and mental health through comprehensive factors such as education, culture, and environment and promoting people's maintenance and improvement of their health. The essential difference between the promotion of physical health promotion and other modes is to emphasize the formation of healthy sports awareness through sports intervention, so as to form a healthy sports lifestyle and improve health. Along with life activities, a variety of information is generated, and various irrelevant information often overlaps [24]. Therefore, in order to detect specific information, it is often necessary to eliminate the interference of irrelevant biological information. Only after acquiring health knowledge, firmly establish the belief of health and persevere. Only in this way can knowledge acquisition be transformed into behavioral change. Comprehensive arrangement should be made to construct the content system of mental health education according to the stages and continuity of individual psychological quality development. It also penetrates into all kinds of school work according to the stage and continuity of individual psychological quality development.

Through the performance of the physical state of the subjects, and the pressures of the subjects before the competition, the main effects of different dimensions of body state under subjects' training are given.

(10) $$\begin{array}{c} \phi_{ij}=\frac{1}{N_{c}}\sum_{\in N_{c}}n_{i}n_{j}. \end{array}$$

The evaluation of the physical state of the body is divided into different stages using physiological and biochemical indicators, which are expressed as

(11) $$\begin{array}{c} F_{ij}^{t}=\frac{1}{N_{c}}\sum_{c\in N_{c}}\frac{f^{t}t_{i}n_{j}}{1+a_{kl}^{c}n_{k}n_{l}}. \end{array}$$

The level of cognition has been improved in both sports practice and theory. Then, use the following formula to calculate the variables of different training factors in the subject's moving image:

(12) $$\begin{array}{c} \sigma_{ij}=\frac{1}{V}\sum_{c\in N_{c}}f_{i}^{c}d_{j}^{c}. \end{array}$$

Two channels of model coefficients corresponding to each level are used as input feature vectors of the respective classifiers. The effect of classifier recognition rate and model order on recognition rate is shown in Tables 4 and 5, respectively. The classifier recognition rate is affected by the quality as shown in Figure 7.

Physical activity is a special social and cultural activity with strong direct participation. Intense competition and frequent interpersonal interactions, as well as diverse forms of activities, are the distinctive features of this cultural event. It is necessary to cultivate people's habits of physical exercise and enhance their awareness of lifelong physical exercise [25]. It is necessary to strengthen the sense of responsibility and ensure the time and effect of physical education classes and daily physical exercise. After health promotion has penetrated into the nonhealth sector, sports have gradually become the main means and means of health promotion. Health promotion is the fundamental way to maintain health. Among them, health maintenance and health promotion strategies are more active mainly because they have a positive meaning of prevention. Bioinformatics is measured on living organisms often in more complex environments. The signal intensity of biological information is generally weak due to the noise interference of biological activities and environmental factors. If an individual feels some obstacles in his past behavioral experience, it will also affect his subsequent behavior. For each individual, each action is accompanied by different feelings, which may be positive or negative. The better the mental health quality, the higher the physical health level.

## 5. Conclusions

Among the cognitive and perceptive factors of sports behavior, perceived sports interests, perceived sports self-efficacy, feelings during sports, and sports social support are significantly positively correlated with regular sports behavior and total exercise volume. The essential attribute and sociological significance of sports determine that sports play a unique role in providing people with social support. Education and exercise are carried out through the interaction between people in sports occasions, which often takes the form of groups. The score of quality of life increased with the duration of exercise. The theory and method of defense and treatment advocated by sports thought will also play an active role in avoiding and getting rid of mental illness for individuals. People's physical and mental health is not optimistic, and sports have a positive effect on people's physical and mental health, and there is a significant correlation between physical health and mental health. College students with proficient sports knowledge have higher quality of life scores than college teachers who do not understand physical exercise knowledge. The quality of life of teachers in the science of exercise is also higher than that of college teachers who are not scientific. Teachers who have lower exercise time and frequency of exercise should also develop a step-by-step exercise program to strive to join them in the sports population.

## Figures and Tables

**Figure 1:** Motion angle data applied to the finite element model.

**Figure 2:** Rotation angle parameters and time relationship.

**Figure 3:** Anaerobic power data index before and after excess recovery.

**Figure 4:** Blood ALP data.

**Figure 5:** Relationship between immediate heart rate and recovery to quiet heart rate before and after the experiment.

**Figure 6:** Maximum exercise capacity data before and after experimental recovery.

**Figure 7:** Classifier recognition rate is affected by quality.

**Table 1:** Peak angle comparison.

Joint name	Male	Female
Hip joint	43.3	41.5
Ankle joint	46.8	42.6
Knee joint	23.6	22.2

**Table 2:** Motion angle parameters applied to the finite element model.

Analysis step	Buckling angle	Adduction angle	Internal rotation angle
1	16.97	9.46	11.44
2	17.35	8.37	10.45
3	13.75	8.68	11.72

**Table 3:** Rotation angle parameters in active and passive situations.

Rotation angle parameters	Healthy side	Ill side
Maximum internal rotation angle	2.58	3.24
Maximum external rotation angle	4.37	3.95
Range of rotation angle	8.96	9.23

**Table 4:** Classifier recognition rate.

(kg)	MLP	SOM
15	81.8	87.8
20	86.7	83.3
25	90.1	82.4

**Table 5:** Influence of model order on recognition rate.

Order of model	15 kg	20 kg	25 kg
3	84.6	86.3	86.4
6	87.5	88.2	89.5
9	88.9	89.5	90.3

## Data Availability

The data used to support the findings of this study are included within the article.
